The article "Increased Asymmetry of Lower Limbs and Leading Joint Angles during Crossing Obstacles in Healthy Male with Cold Exposure" was published in 2022. Journal: Appl Bionics Biomech.

# Increased Asymmetry of Lower Limbs and Leading Joint Angles during Crossing Obstacles in Healthy Male with Cold Exposure

**DOI:** 10.1155/2022/6421611

**Published:** 2022-10-15

**Authors:** Shun Yao, Yu Su, Yu-Hong Jiang, Tze-Huan Lei, I-Lin Wang, Shang-Lin Hsieh

**Affiliations:** ^1^Jilin Sport University, No. 2476, Freedom Road, Nanguan District, Changchun City, 130022 Jilin Province, China; ^2^College of Physical Education, Hubei Normal University, Huangshi, China; ^3^Health Technology College, Jilin Sport University, Changchun, 130022 Jilin, China; ^4^M.D Orthopedic Department, China Medical University Hospital, Taichung, Taiwan

## Abstract

Lower ambient temperatures impair neuromuscular function and balance. However, whether lower ambient temperatures could alter joint angles and symmetry of lower limbs during crossing obstacles in males still remains unknown. Therefore, we investigated whether there is reduction of ambient temperature (20°C; 15°C; 10°C) on lower limbs joint angles and symmetry when crossing obstacles in males. On three different occasions, eighteen male participants underwent 30 min exposure to three different environmental temperatures (10°C, 15°C, and 20°C), which was followed by the obstacle crossing test at 10%, 20%, and 30% of the participant leg length. In each trial, we assessed joint angles and symmetry of lower limbs when crossing obstacles at 10%, 20%, and 30% of the participants' leg length. The results showed that leading limb maximum joint angles were greater in 10°C than in 15°C and 20°C when leading limb crossed obstacle heights of 20% and 30% leg length (*p* < 0.05). Trailing limb maximum joint angles were not different (*p* > 0.05). Lower limb asymmetry increased when participants crossed obstacle heights of 20% and 30% leg length at 10°C (*p* < 0.05). This study concluded that in male participants, cold exposure can increase lower limb asymmetry to increase falling risk when crossing obstacles. Also, the increased leading limb joint angles and constant trailing limb joint angles increase safety during crossing obstacles.

## 1. Introduction

Death and disease caused from cold have become a major public health problem. Previous study has showed that the body can lose heat faster than it is produced in cold weather, which led to hypothermia [1]. Hypothermia can increase the incidence of fall-related hip fractures and many types of musculoskeletal diseases, including lower back pain, tenosynovitis, carpal tunnel disease, and so forth. [2, 3]. Therefore, a cold environment may be a factor that increases body damage. In addition, cold exposure can aggravate pain in damaged joints and interfere daily activities [4]. Human concentration and vigilance were reduced in cold environments to increase accidents and injuries in occupational and leisure activities [5]. Therefore, cold exposure may damage human health and affect daily activities in multiple ways.

Overcoming obstacles is an essential and complex part of daily activities. Compared with walking, increased swing limb elevation during obstacle crossing increases the balance demands [6]. Decreased balance will increase the risk of falling and lead to body injury during walking [7]. Therefore, maintaining effective body control of postures can ensure safety while crossing obstacles. However, previous study has shown that cold exposure impairs postural control by affecting a variety of mechanisms [5]. Cold exposure could reduce the acuity of sole and ankle mechanoreceptors or the proprioceptors located in the muscles, tendons, and joints and affect postural control [5]. Cold exposure could also slow down neural transmission, making fine-tuning more difficult and increasing risk of falling [8]. Therefore, cold exposure may alter the stability of the body to increase the risk of falling and body injury while crossing obstacles.

Gait involves a cyclical and laterally alternating progression from an unsteady balance during the single limb stance phase to a quasistable balance during the dual limb stance phase [9]. Slight asymmetry of the gait may reflect functional differences in the contribution of each limb to propulsion and control during walking [9]. Therefore, symmetry becomes an important healthy feature of gait [10]. In addition, gait symmetry is associated with stabilization of postural control during walking [10]. However, cold exposure may alter the stability of the body to reduce gait symmetry while crossing obstacles. Previous studies have not explored the effect of cold exposure at different temperatures on lower limb symmetry in men when crossing obstacles. Therefore, the purpose of this study is to investigate the effect of decrease in ambient temperature (*T*_amb_) (20°C, 15°C, and 10°C) on lower limb symmetries and joint angles when crossing obstacles in males. We hypothesized that leading limb joint angles and lower limb asymmetry would increase when crossing obstacles at 10°C than 15°C and 20°C.

## 2. Materials and Methods

### 2.1. Participants

Eighteen healthy male participants were recruited (age: 21.7 ± 0.9 years, height: 178.5 ± 5.4 cm, mass: 72.4 ± 9.7 kg). All participants had no neuromusculoskeletal dysfunction or musculoskeletal issues, resulting in abnormal gait. Furthermore, all participants were required to abstain from alcohol or coffee and intensive physical exercise 48 h prior to testing. This study was approved by Jilin Sports University (IRB NO: JLSU-IRB2020007) and performed in accordance with the Declaration of Helsinki.

### 2.2. Experimental Design

All participants were needed to complete three *T*_amb_ trials, including (1) 20 ± 0.5°C; (2) 15 ± 0.5°C; (3) 10 ± 0.5°C to evaluate the effects of lower ambient temperatures on lower limb joint angles and symmetry when crossing obstacles. All of the trials were randomized, counter-balanced, and separated by 48 h apart. In order to avoid the influence of the diurnal rhythms on body temperature fluctuation, all trials were performed in the morning between 8 A.M. and 11 A.M.

### 2.3. Protocol

Before the *T*_amb_ trial, participants' leg lengths were measured. Then, they familiarized themselves with the walkway and by crossing three obstacle heights: 30%, 20%, and 10% leg lengths to adjust their starting position to ensure the correct limb to cross the obstacle. Following that, participants wearing uniform shorts and shoes entered the laboratory to get started with whole-body cold exposure. The environmental conditions were required to be kept constant and controlled at a humidity of 35 ± 5% and the air velocity less than 0.2 m·s^−1^. Participants needed to sit quietly in a chair and expose themselves to three different *T*_amb_ for 30 min. The choice of 10–20°C as the environmental control temperature range is based on the most relevant research and commonly experienced temperature range in daily life [11]. After whole-body cold exposure, the experimenter completed the reflective marker taping within 2 min. Then, participants walked at a self-selected speed to cross the height-adjustable obstacles on the walkway. The *T*_amb_ during the participant walking was as the same as *T*_amb_ during cold exposure. All subjects were required to use the left and right legs as leading limbs to cross obstacles at three ambient temperatures. The leading limb was defined as the leg that crosses the obstacle first [12]. There were three successful ambient temperature trails, and each trail had three conditions: (1) crossing obstacles at a height of 30% of the leg length, (2) crossing obstacles at a height of 20% of the leg length, and (3) crossing obstacles at a height of 10% of the leg length. All conditions were randomized and counter-balanced.

### 2.4. Data Collection

Two infrared reflective markers were placed on either ends of the tube to define the position of the obstacle. A modified Simple Helen Hayes with 19 reflective markers was secured over selected anatomic landmarks to track the motion of the body segments (as previous research [13]). A 10-camera system (Vicon V5 cameras, Vicon Motion Systems Ltd., Oxford, UK) and Nexus software (Version 2.9.0, Vicon Motion Systems, UK) were used to capture the motion with a sampling rate of 200 Hz and a fourth-order Butterworth filter with a cut-off frequency of 5 Hz for low-pass filtering, while three force plates (AMTI BP600900) were used at a sampling frequency of 1200 Hz to collect ground reaction forces (GRF). The 1st and 3rd plates collected GRF before and after the trailing limb crossed the obstacle; the 2nd plate collected GRF after the leading limb crossed the obstacle.

### 2.5. Data Analysis

All the data files were imported and processed under MATLAB (R2019a, The MathWorks, Natick, USA). Markers data for each trail condition were used to calculate the maximum left/right leading joint angle and the maximum left/right trailing joint angle. Maximum left/right leading joint angles were defined as the maximum joint angles of the left or right leading leg from the toe above obstacle to landing. Maximum left/right trailing joint angles were defined as the maximum joint angle of the left or right trailing leg from landing to toe-off. Five gait spatiotemporal parameters (*V*), step length, swing time, stance time, double support (DS) time, and swing time, to the standing time ratio (SW/ST) were calculated (Figure 1). Five gait spatiotemporal parameters were used in the equation to explore the lower limb asymmetry. The equation is as follows:

(1) $$\begin{array}{c} \text{Gait asymmetry }\left(\text{GA}\right)\text{: GA}=100*\text{Ln}\left[\left(\frac{V_{\text{leading}}}{V_{\text{trailing}}}\right)\right]. \end{array}$$

Equation (1): Ln is the logarithm to the base of the mathematical constant.

### 2.6. Statistical Analysis

All statistical analyses were performed in MATLAB software. The experiment used repeated measures two-way analysis of variance (ANOVA) (*T*_amb_ × obstacle height). When the interaction was found to be significant, post hoc comparisons were made using Bonferroni multiple comparisons. The significance level was set at *P* < 0.05. The modified Cohen scale is used to determine the size of the three drop height variations, <0.2 means slight difference, 0.2–0.6 means small difference, 0.6–1.2 means medium difference, and 1.2–2.0 large difference [14].

## 3. Results

The ambient temperature of 10°C affected maximum leading joint angles and the lower limb symmetry, as assessed by obstacle crossing. In particular, the maximum leading joint angles and lower limb asymmetry were greater in 10°C than in 15°C and 20°C.

Figure 2 illustrates that significant interactions between *T*_amb_ and the obstacle height were observed in the maximum left and right leading joint angles of the ankle, knee, and hip (left/right ankle: *p* = 0.046, *p* = 0.020; left/right knee: *p* = 0.027, *p* = 0.018; left/right hip: *p* = 0.001; *p* = 0.001). Furthermore, the post-hoc analysis showed that the maximum leading joint angles of the ankle, knee, and hip were greater in 10°C than in 15 °C and 20 °C when the left and right leading limbs crossed obstacle heights of 20% and 30% leg length (all *p* < 0.001, ES = 0.84–3.73). However, there were no significant differences when the left and right leading limbs crossed an obstacle height of 10% leg length.  Figure 3 also presented that there were no significant interactions between *T*_amb_ and the obstacle height in the maximum trailing joint angle (all *p* > 0.05). The *T*_amb_ and obstacle height also did not exhibit significant main effect, as shown in Figure 3 (all *p* > 0.05).

Figure 4 illustrates that significant interactions between *T*_amb_ and obstacle height were observed in swing time GA, stance time GA, and SW/ST GA (left/right swing time GA: *p* = 0.008, *p* = 0.044; left/right stance time GA: *p* = 0.043, *p* = 0.008; left/right SW/ST GA: *p* = 0.001; *p* < 0.001). Compared with 15°C and 20°C results, the 10°C results showed a significant increase in swing time GA, stance time GA, and SW/ST GA when the left and right leading limbs crossed obstacle heights of 20% and 30% leg length (all *p* < 0.001, ES = 0.44–0.75). However, there were no significant differences when the left and right leading limbs crossed an obstacle height of 10% leg length. Figure 4 also presented that there were no significant interactions between *T*_amb_ and the obstacle height in step length GA and DS time GA (All *p* > 0.05). At the same time, there are no significant *T*_amb_ and obstacle height main effect (All *p* > 0.05).

## 4. Discussion

The purpose of this study was to investigate whether lower ambient temperatures could alter joint angles and symmetry of lower limbs when crossing obstacles in males. The results showed that leading limb joint angles and lower limb asymmetry increased in 10°C than in 15°C and 20°C when participants crossed obstacle heights of 20% and 30% leg length. Our results agreed with our study hypothesis where the reduction of ambient temperature would increase the leading limb joint angles and lower limb asymmetry during obstacle crossing. This therefore indicates that the drop in ambient temperature may increase the risk of falling in male when crossing obstacles.

The leading limb was raised with increasing ankle, knee, and hip joints angles to ensure safety and avoid falls when crossing obstacle heights of 20% and 30% leg length, whereas there were no changes at 10% leg length height. Previous study has shown that body exposed to cold environments can decrease lower limb muscle strength to increase risk of falls [15]. The toe-clearance affects the safety of crossing the obstacle, while increased leading toe-clearance helps reduce the risk of tripping [16]. The toe-clearance depends on hip and knee joint flexion and ankle dorsiflexion [17]. The swinging limbs would increase the ankle, knee, and hip joints angles to be raised to increase toe-clearance in order to prevent falling and ensure safety when crossing obstacles [16, 18, 19]. In this study, exposure to cold at 10°C ambient temperature may reduce muscle strength and increase the risk of falling, the lower limbs raise the leading limb with increasing ankle, knee, and hip joints angles to reduce the risk of falls, thus ensuring safety when crossing obstacles at 20% and 30% heights.

The maximum ankle, knee, and hip joints angles of the left and right trailing limbs did not change when crossing obstacle heights of 30%, 20%, and 10% leg length at 10°C compared to 15°C and 20°C. The joint angles remained unchanged during the maximum trailing period, which may be for maintaining the dynamic stability of the body when the leading limbs cross obstacles. Previous study has pointed out that the trailing limbs can support the body when stepping over obstacles with the leading limbs [20]. The lower limbs are in a closed kinematic chain state during the stance phase of walking and the stability of the trunk rely on the stability provided by the distal segment of supporting limbs [21]. In this study, the angles of the trailing limbs joints did not change during the maximum trailing period at 10°C to maintain their own stability. In addition, the soles of the trailing limb can receive sensory feedback from cutaneous receptors and transmit them to the central nervous system [22]. The central nervous system will precisely control the trailing limb position to reduce the possibility of trailing limb contact with obstacles to decrease the risk of tripping [23, 24]. In summary, the body may be precisely controlled by the central nervous system to keep the trailing limb position unchanged so as not to change the maximum joint angle of the trailing limb, thus increasing its stability to further reduce the falling risk when crossing obstacles at 10°C.

The swing time GA, stance time GA, and SW/ST GA between leading and trailing limbs increased when crossing obstacle heights of 20% and 30% leg length, except for 10%, at 10°C than 15°C and 20°C. However, there is no significant difference in step length GA and DS time GA when crossing obstacle heights of 30%, 20%, and 10% leg length at 10°C compared to 15°C and 20°C. The body's reduced balance in a cold exposure environment may disturb gait stability and increase bilateral asymmetry between the leading and trailing limbs, thereby increasing the risk of falls. Previous study has pointed to an increase in swing time GA as an important marker of reduced balance during walking [25]. Decreased gait stability can cause increased swing time GA [26] and may be caused by a severe decrease in neuromuscular strength [27]. Therefore, in the present study, the increase in swing time GA between the leading and trailing limbs over obstacle heights of 20% and 30% leg length at 10°C ambient temperature may be due to a decrease in lower limb muscle strength caused by cold exposure, resulting in gait stability impairment. In addition, cold exposure inhibits the acuity of cutaneous receptors on the feet soles and joints proprioceptors, slowing muscles nerve conduction and impairing the body's balance [8, 28, 29]. The body instability can lead to an increase in stance time GA [30]. Therefore, the decrease in sensory transmission capacity at 10°C ambient temperature may cause reduced the body dynamic stability and increased stance time GA when the lower limb crossed a higher obstacle height. Accordingly, swing time, stance time, and SW/ST ratios were highly positively correlated [10]. In this study, the increase in SW/ST GA at 10°C was caused by the increase in swing time and stance time.

There are still some limitations of this study. First of all, this study did not collect changes in body blood biochemical data to reflect the impact of different environmental temperatures on body function. Second, this study did not measure the EMG parameters of the lower limbs related muscles. Cold exposure could impair muscle performance. EMG parameters may reflect lower limbs muscle performance to illustrate the effects of cold exposure. Therefore, this issue deserves further study.

## 5. Conclusions

This study suggests that lower ambient temperature can increase leading limb joint angles and lower limbs asymmetry when participants crossed obstacles heights of 20% and 30% leg length, resulting in a decrease in postural stability and an increase in falls over obstacles. The bilateral asymmetry between the leading limb and trailing limb increased under lower temperature environment with higher risk of falling. Men may increase their fall risk after cold exposure and take more conservative strategies to reduce the fall risk and achieve safer obstacle crossings. This study is helpful to warn people who live or work in cold environment that they should keep themselves warm in such cold conditions to prevent the decrease in balance and the increase in limb asymmetry, which lead to the increase of the falling risk; it is also necessary to improve muscle strength and proprioceptive sensitivity to reduce the incidence of falls.

## Figures and Tables

**Figure 1:** Schematic diagram of leading and trailing limb gait spatiotemporal parameters.

**Figure 2:** Maximum ankle angle (a) and (b), knee angle; (c) and (d), and hip angle; (e) and (f) of the left and right leading limbs changed when crossing obstacle heights of 10%, 20%, and 30% leg length (10% LL; 20% LL; 30% LL) at three different *T*_amb_ (20°C; 15°C; 10°C). “∗” significant *T*_amb_ × height interaction effects (*p* < 0.05). “‡” indicates a significant difference in 10°C compared with 20°C. “†” indicates a significant difference in 10°C compared with 15°C.

**Figure 3:** Maximum ankle angle (a) and (b), knee angle (c) and (d), and hip angle (e) and (f) of the left and right trailing limbs did not change when crossing obstacle heights of 10%, 20%, and 30% leg length (10% LL; 20% LL; 30% LL) at three different *T*_amb_ (20°C; 15°C; 10°C).

**Figure 4:** Step length GA: (a) and (b) swing time GA; (c) and (d) stance time GA; (e) and (f) DS time GA; (g) and (h) and SW/ST GA; (i) and (j) between leading and trailing changed when crossing obstacles height of 10%, 20%, and 30% leg length (10% LL; 20% LL; and 30% LL) at three different *T*_amb_ (20°C; 15°C; and 10°C). “∗” Significant *T*_amb_ × height interaction effects (*p* < 0.05). “‡” indicates a significant difference in 10°C compared with 20°C. “†” indicates a significant difference in 10°C compared with 15°C.

## Data Availability

The data results are included in the manuscript.

## Abbreviations

*T*_amb_: Ambient temperature
GRF: Ground reaction forces
DS: Double support
SW/ST: Swing time to standing time ratio
GA: Gait asymmetry.
